# Phytotoxicological study of selected poisonous plants from Azad Jammu & Kashmir

**DOI:** 10.1371/journal.pone.0263605

**Published:** 2022-05-11

**Authors:** Faisal Rasool, Zaheer Ahmed Nizamani, Khawaja Shafique Ahmad, Fahmida Parveen, Shahzad Akbar Khan, Naveed Sabir

**Affiliations:** 1 Department of Veterinary Pathology, Faculty of Animal Husbandry and Veterinary Sciences, Sindh Agriculture University, Tandojam, Pakistan; 2 Department of Pathobiology, Faulty of Veterinary and Animal Sciences, University of Poonch Rawalakot (UPR), Azad Jammu & Kashmir, Pakistan; 3 Department of Botany, University of Poonch Rawalakot (UPR), Azad Jammu & Kashmir, Pakistan; Mirpur University of Science and Technology, PAKISTAN

## Abstract

Poisonous plants cause tremendous economic losses to the livestock industry. These economic losses are deterioration in their health, decreased productivity, deformed offspring, and reduced longevity. The current study is the first comprehensive report on poisonous plants of Azad Jammu and Kashmir which systematically documents the phytotoxicological effect and mode of action in livestock. The information was gathered from 271 informants including 167 men and 104 women through semi-structured interviews and literature search through available databases. The data collected through interviews was analyzed with quantitative tools viz. the factor informant consensus and fidelity level. A total of 38 species of flowering plants belonging to 23 families and 38 genera were reported. Family Asteraceae (5 spp) was the most dominant, followed by Solanaceae (4 spp), Fabaceae (4 spp), Euphorbiaceae (4 spp) and Convolvulaceae (3 spp). Among all the species collected, herbs were the dominant life form (22 spp, 57.89%), trailed by shrubs (11 spp, 28.95%), and trees (5 spp, 13.16%). Whole plant toxicity was reported to be the highest (15 spp, 39.47%), followed by leaf toxicity (12 spp, 31.58%), seed toxicity (4 spp, 7.89%), fruit toxicity (3 spp, 10.53%), latex toxicity (2 spp, 5.26%), flowers toxicity (1 spp, 2.63%), and berries toxicity (1 spp, 2.63%). The most toxic route of administration was found oral (39 spp, 40.63%), followed by intraperitoneal (24 spp, 25%), and intravenous (21 spp, 21.88%). The most commonly affected organ was found liver (20.41%), followed by gastrointestinal tract (20.341%), CNS (16.33%), skin (14.29%), kidneys (12.24%), lungs (4.04%), reproductive organs (2.04%), spleen (1.75%), blood (1.75%), heart (1.75%), urinary tract (1.75%), and pancreas (1.75%). The maximum *F*_ic_ value was found for dermatological disorders (0.91), followed by the endocrine system (0.90), gastrointestinal (0.82), neurology (0.77), nephrology (0.67), cardiovascular (0.67), urinary (0.67), respiratory (0.60), sexual (0.60) disorders. *Senecio vulgaris*, and *Ageratum conyzoides* were the most important plants with fidelity level (0.95) and (0.87). *Nerium oleander*, *Lantana camara*, *Leucaena leucocephala*, and *Ricinus communis* were the important poisonous plant with maximum fidelity level (100%). *Ricinus communis* with reported lowest LD_50_ (<20 mg/kg) was the top-ranked poisonous plant followed by *Lantana camara* and *Justicia adhatoda* (25–50 mg/kg), *Nerium Oleander* (157.37 mg/kg), and *Datura innoxia* (400 mg/kg). We found that knowledge about poisonous plants is less prevailing in the rural areas of Azad Kashmir compared to the knowledge about medicinal plants and poisonous nature of reported plants is due to production of toxic substances and presence of essential oils.

## Introduction

The livestock industry suffers huge economic losses as a result of poisonous plants [1, 2]. These economic losses are caused by a decline in their health, decreased output, abnormal progeny, and decreased lifespan [3]. Animals encountering poisonous plant may show different kinds of symptoms e.g., irritation of skin by contact [4], internal poisoning by ingestion [5], absorption by the dermal layer [6], and inhalation through respiratory system [7].

Toxic plants are classified into groups based on their poisonous properties [8]. Within a single genus or family, these principles are chemically similar or identical, especially if the taxa are closely related [3]. Animals are often affected accidently by poisonous plants because of drought season and over grazing in pastures, [9, 10] and lack familiarity of potential toxic plants by nomads and villagers during hay feeding [11]. Many factors determine plant toxicity in livestock, including amount and number of plants eaten, plant growth conditions and flowering stage [12].

Among livestock, intensity of plant toxicity can vary with species, age, sex, and general body condition [13]. The most important reason for livestock exposure to plant poisoning is shortage of feed and nutrition and sudden exposure to plants [14]. Shortage of food forces animals to browse those plants which are well documented to have high level of toxic metabolic compounds [15], causing loss in productivity, illness, and death in animals [16]. The nature of the toxic secondary metabolites varies with respect to place of origin and surrounding environmental conditions [17]. The key substances in plant which function against herbivores in plant defensive system are tannins [18] phenolics [19], alkaloids [20], phytohemagglutinins [3], terpenes [21], cyanogenic glycosides [22], and oxalates [23].

The key toxins present in plants may cause severe diseases in livestock resulting in huge economic losses every year. For example, phytotoxin racin of *Ricinus communis* cause anorexia, apathy, dyspnea, abdominal cramps, piloerection, abortion, acute purgation, and gastrointestinal irritation [24], lantadenes of *Lantana camara* trigger hepatotoxicity, chronic cholestasis, piloerection, and photosensitization [25]. Likewise, Oleandrin of *Nerium oleander* cause piloerection, abdominal salivation, vomiting, diarrhea, irregular heartbeat, drowsiness, tremors, seizures, coma, hepatotoxicity, and nephrotoxicity [26]. The principal toxin cicutoxin of *Leptopus cordifolius* is responsible for muscle weakness, piloerection, bone lesions, aneurysms, and burning sensation [27], scopolamine and hyoscyamine of *Datura stramonium* are responsible for dermatitis, polydipsia, mydriasis, anorexia, abdominal pain, stupefaction, restlessness [28].

Poisonous plants that cause various maladies have been reported in previous studies [15, 29–32], as well as the numerous compounds present in them that cause toxicity. Anxiety, panic reactions, and psychiatric symptoms are the most common clinical side effects, all of which are frequently reported by novice users [33]. The potent poisonous components, which may be delivered in very small amounts into the body of animal, will have a detrimental effect and may be deadly at times [30, 34]. These poisonous compounds cause damage to the cell’s protoplasm, with immediate or progressive consequences [3], and their quantity fluctuates with seasonality and plant type [35].

Plant toxicity science is developing day by day with emergence of new methodologies, with the development of methods, ideas, and insight. A little attention has been paid so far on poisoning caused by compounds present in plants, thus the mode of action of plant poisoning remains largely unknown. Plant poisoning is more or less owing to unintentional consumption of seeds, fruits, pollens, trichomes, and other plant parts [36]. Toxic plants have the potential to harm every organ system and endanger animal health and productivity. There are hundreds of plant species in the field that might create animal toxicity problems. It is critical to become familiar with these plants, their toxicity mechanisms, and consequences. By careful study of literature, it is quite clear that up till now, there is no such study for identification and characterization of native poisonous plants in Azad Jammu and Kashmir. Moreover, the toxicity level of these plants has also not yet been assessed through nomads and other livestock rearer. The present study thus has been designed to fill the existing gaps of research by identification of poisonous plant and by determining their toxicity level.

## Material and methods

### Ethics statement

The study was approved by the “Institutional Ethics Committee of Sindh Agriculture University Tandojam” through No. SAUT/ASRB/VP/1280. Verbal informed consent was obtained from each informant before conducting the interview process.

### Study area

The State of Azad Jammu and Kashmir (AJK) lies between 33.9259° N, 73.7810° E and has a total area of 13,297 km^2^ (Fig 1). The AJK has a subtropical to temperate climate due to its altitudinal range of 600–2900 meters above mean sea level [10]. The research site’s yearly temperature ranges from 21°C in the summer to 1.0°C in the winter, with an average rainfall of slightly more than 1551 mm [37]. Maize, wheat, rice, and millet are the main crops farmed in AJK, while grains, pulses, oilseeds, and vegetables are minor crops. Maize is farmed in a variety of agro-ecological zones at an elevation ranging from 1,828 meters to 3,656 meters [38].

**Fig 1:** Map of the study area showing study sites in all district of Azad Jammu and Kashmir. (Source: https://www.ajk.gov.pk/ajkmap).

### Plant collection and preservation

A detailed survey was conducted on poisonous plants which cause toxicity in small ruminants of AJK. A total of 271 volunteer individuals belonging to different professions were interviewed from March to November 2019–2020 using semi structured questionnaires (Table 1). The informants selected through snowball method were of different ages (20–80 years old) and professions i.e., veterinary doctors, veterinary assistants, artificial inseminator, livestock assistant, lab technicians, agriculturist officer, farmer, cattle attendant, domestic cattle and buffalo holder, and nomads. Informed consents were obtained from each informant prior to start interviews and the Code of Ethics of the International Society of Ethnobiology was followed. For interviews, semi-structured questionnaires were first developed in English and later translated into different languages (Urdu, Kashmiri, Hinko, Pahari, Pothohari, Gojri, Balti, Shina, Saraiki, Punjabi, and Sindhi) with the help of translators [39]. The information collected was focused on nature of plant, parts of plant eaten, toxicity level, animal type affected, seasonality, major symptoms, animal sex and age, first and second animal symptom appearance, abortion, nature of disease (specific / common), morbidity and mortality ratio [37]. During the interviews, qualitative ethnographic data was documented following Iqbal et al. [40] and Alexiades and Sheldon [41]. The poisonous plants found in the research region were collected and identified using the Flora of Pakistan [42], with names confirmed by literature (www.efloras.org/index.aspx) and the Kew grass database (https://www.kew.org/data/grasses-db/index.htm). Standard herbarium protocols were followed strictly for the voucher specimen [43, 44]. For reference purposes, the plants were catalogued and stored in the Department of Botany, University of Poonch Rawalakot Herbarium (Fig 2).

**Fig 2:** Pictorial view of some highly poisonous plants based on their LD50 values and respondent scores. a. *Nerium oleander*, b. *Ricinus communis*, c. *Leptopus cordifolius*, d. *Justicia adhatoda*, e. *Datura stramonium*, f. *Dodonaea viscosa*, g. *Lantana camara*, h. *Euphorbia helioscopa*, i. *Solanum surattense*.

**Table 1:** Demographic characteristics of the informants selected from the study area.

Variable	Demographic category	Numbers	Percentages
Gender	Male	167	61.62
	Female	104	38.38
Age	20- 30Years	67	24.72
	31–40 Years	102	37.64
	41–50 Years	69	25.46
	51–60 Years	17	6.27
	60–80 Years	16	5.90
Occupation	Veterinary doctors	49	18.08
	Traditional practitioners (TP)	56	20.66
	Veterinary assistants	13	4.80
	Artificial inseminator	19	7.01
	Livestock assistant	13	4.80
	Lab. technicians	21	7.75
	Agriculturist officer	13	4.80
	Farmer	15	5.54
	Cattle attendant	11	4.06
	Domestic cattle and buffaloes holder	21	7.75
	Nomads	17	6.27
	Domestic goat and sheep holders	23	8.49
Literacy Level	Illiterate	167	61.62
	Primary	55	20.30
	Middle	16	5.90
	Intermediate	13	4.80
	Graduate	7	2.58
	Master	5	1.85
	M.Phil.	5	1.85
	PhD	3	1.11

### Informant consensus factor (FIC)

The factor informant consensus (Fic) was used to identify plants with special intercultural significance, as well as the agreement for plants that cause livestock diseases [45, 46]. The numerous ailments induced by poisonous plants were divided into major categories [45]. If plants are picked at random or informants do not share knowledge about their participation in causing toxicity in cattle, Fic values are low (around 0). If there is a well-defined selection criterion in the community and/or if information is transmitted amongst informants, values were high (around 1) [46–48]. The Fic was calculated as the number of citations in each category (nur) minus the number of species identified for toxicity (nt), divided by the number of use citations in each category minus one [45].


$$ICF=1+\frac{nur-nt}{nur-1}$$

### Fidelity level (Fl)

The fidelity level (Fl) was calculated for the most frequently reported diseases or ailments. It is the ratio between the number of informants who independently suggested the role of a species for poisoning and the total number of informants who mentioned the involvement of plant poisoning in livestock [49].


$$FL=\frac{Np}{N}\times 100$$

Where Np is the number of informants who claimed about plant poisoning responsible for a particular ailment in livestock, and N is the number of informants who experienced plant poisoning that caused symptoms or sign of disease in their livestock [49, 50].

### Literature survey

To develop a broader picture of their previously reported pharmacological activities and cross-examining the toxicity of plants, information was retrieved from scientific databases such as PubMed, Scifinder, Google Scholar, ScienceDirect, Scopus, Chemical Abstracts Services, books, dissertations, and technical reports contained in the libraries of the University of Poonch Rawalakot AJK, and NAPRALERT. The search engines employed the terms Azad Jammu and Kashmir, ethno-veterinary, poisonous plants, toxicity, and livestock as keywords. To find relevant information, researchers who were undertaking ethno-veterinary research in Azad Jammu and Kashmir were consulted. The search was conducted initially in March to November 2019–2020 as part of a PhD dissertation [51]. An inclusive exploration commenced by all the earlier investigation in last 40 years (1981–2021) in different regions of the world was reviewed. During this process, we gathered all the information regarding adverse effect of poisonous plant on livestock health. [37]. Individually in each paper, the data regarding botanical names of plants used, family, local name, plant life form, poison plant parts, indication or disease treated, animal/ livestock species affected, dosage and level of toxicity (LD_50_), mode of action, toxin responsible, clinical lesions, mode of administration, affected organs, suspected species, and breeds was collected. To avoid biasness and misinterpretation, we used information extracted from the informants and available in the literature.

## Results

### Demography

A total of 271 informants, including 167 men and 104 women were interrogated to extract the local knowledge on plant poisoning in livestock in different parts of AJK. These included veterinary doctors, veterinary assistants, artificial inseminator, livestock assistant, lab technicians, Gujjar’s/farmer, Bakkarwals (nomads), veterinarians, livestock rearers, dairy owners, milkmen, traditional practitioners, and agricultural experts. The traditional practitioners and veterinary doctors were all men. The informants age group ranged between 20 and 80 years. About, 61.62% informers were uneducated, and rests were educated up to master and PhD level.

### Floristic contribution

In this study, a total of 38 poisonous plant species belonging to 23 families and 38 genera were reported (Table 2, Fig 3). The most common family was Asteraceae (5 species), which was followed by Solanaceae (4 species), Fabaceae (4 species), Euphorbiaceae (4 species), and Convolvulaceae (4 species) (3 spp). Only one species represents each of the eighteen families (Fig 3). Herbs (Fig 4) were the most common life form (22 spp, 57.89%), followed by shrubs (11 spp, 28.95%), and finally trees (11 spp, 28.95%). (5 spp, 13.16%).

**Fig 3:** Distribution of poisonous plants in different families.

**Fig 4:** Percentage of distribution of poisonous plant different plant functional types (PFTs).

**Table 2:** List of poisonous plants with their botanical names, toxic plant parts, route of administration and signs.

S. No	Family	Botanical name	Local name	Habit	Toxic plant part	Susceptible species /Breed	Affected organ /system	Mode of administration	Clinical signs
1	Amaranthaceae	*Achyranthes aspera* L. (Poonch 126)	Puthkanda	Herb	Wp	Rats, mice	CNS	IV, IP, oral	Anorexia, acute purgation, weight loss, reduced food and water intake, poor response to external stimuli, drowsiness, lethargy, piloerection of hair, paddling of feet, sluggishness
2	Asteraceae	*Ageratum conyzoides* L.	Neeli jari	Herb	Wp	Rats, humans, mice, rat, guinea pigs, rabbits and dogs	Heart, liver, kidney	Oral	Severe itching, shivering, anorexia, very high fever, production of bitter milk, anorexia, intense diarrhea, and death.
3	Araceae	*Alocasia indica* (Lour.) Spach	Lambapatar	Herb	Leaves	Rats, mice	Liver, testis,	Oral	Infertility in mice, hepato-renal disorder, weight loss, sperm abnormalities, reduced LH & FSH levels.
4	Primulaceae	*Anagallis arvensis* L.	Kokoon	Herb	Wp	Rat, mice, calves, sheep	Kidney, gastrointestinal tract	IP, oral	Headache, nausea, dyspnea, anorexia, excessive thirst, trembling of limbs, general weakness, inability to stand with head hanging down and ears drooping, hypothermia, dysentery, unconsciousness and ultimately death
5	Papaveraceae	*Argemone mexicana* L.	Peeli kandiari	Herb	Seeds	Rat, mice	CNS	Oral, Intragastric.	Sedation, sluggishness, muscular jerks, abdominal contractions and increased defecation, black secretions from the eyes, piloerection, oedema of the hind legs and submandibular and mortality. Weight loss, headache, nausea, vomiting, diarrhea
6	Fabaceae	*Bauhinia variegata* L.	Kachnar	Tree	Leaves	Rat, mice	GIT	Oral	Changes in behavior of rat, Monocytes and lymphocytes decreased at high doses.
7	Asteraceae	*Bidens bipinnata* L.	Kandili jari	Herb	Fruit	Mice, chicken	GIT	Oral	Irritation of throat, hepatitis
8	Asclepiadaceae	*Calotropis procera* Aiton	Desi aak	Shrub	latex	Rat, mice, rabbit	Liver, intestine, heart, spleen,	Oral,	Convulsion, diarrhea, dyspnea, alopecia, bradycardia, frothy vomiting, photophobia, irritant to skin and blisters on mucous membrane, eyes inflammation, drastic purgation, and abortion in pregnant animals
9	Cannabinaceae	*Cannabis sativa* L.	Bhang	Herb	Wp	Companion animals and human	CNS	Oral	Narcotic and sedative whose intake (either in fresh or dry state) causes nausea, vomiting, mydriasis, excitement, hallucination, anorexia, drowsiness, delirium, and stupefaction
10	Ranunculaceae	*Clematis grata* Wall	Bail	Shrub	Leaves	Cattles, dog, cat,	Lungs	Oral, inhalation, dermal	Salivation, slight vesication, weakness, respiratory difficulty, nausea, convulsions, coma, death
11	Apiaceae	*Conium maculatum* L.	Shokra	Herb	Wp	Cattle, sheep, goat, horses, Pigs poultry, turkeys, quails and monogastric animals	CNS	Oral, IM	Vomiting, trembling, problems in movement, slow, Appetites, slobber, rapid pulse, rapid respiration, bloat rapid feeble pulse. Muscular incoordination severe pain, salivation, urination, nausea, convulsions, coma and death.
12	Convolvulaceae	*Convolvulus arvensis* L.	Hiran khuri	Herb	Wp	Humans, animals, mice, rat, rabbits, dogs	GIT	IV, IP, oral	Drastic purgative, gastrointestinal irritation, diarrhea, urogenital disorders, and animal stings
13	Cuscutaceae	*Cuscuta reflexa* Decne.	Kaandal	Herb	Wp	Cattle, sheep, goat, horses, Pigs poultry turkeys	GIT	IV, IP, oral	Uneasiness, vomiting, anorexia, abdominal pain, purgation, abortion
14	Fabaceae	*Dalbergia sissoo* Roxb	Tali	tree	Leaves	Sheep, goat, rat	Reproductive system	IV, IP, oral	Abortion in animals
15	Thymelaeaceae	*Daphne oleoides* Schreb.	Kaagi sadi	Shrub	Leaves	Humans, mice, rat, rabbits, dogs	Skin	IV, IP, oral	Nausea, vomiting, burning sensation in mouth, restlessness, stupor, severe diarrhea, loss of consciousness
16	Solanaceae	*Datura innoxia* Mill	Datura	Herb	Leaves	Sheep, goat, rat	Skin	IV, IP, oral	Dermatitis, dryness of mouth and throat, polydipsia, mydriasis, anorexia, abdominal pain, stupefaction, restlessness
17	Solanaceae	*Datura stramonium* L.	Datura	Herb	Wp	Humans, mice, rat, rabbits, dogs	CNS	IV, IP, oral	Fruits are sedative. piloerection accidental intake of seeds or leaves by livestock causes drowsiness, dryness of mouth and throat, blurred vision, mydriasis
18	Sapindaceae	*Dodonaea viscosa* Jacq.	Sanatha	shrub	Leaves	Sheep, goat, rat	Stomach	IV, IP, oral	Nausea, vomiting, shivering
19	Euphorbiaceae.	*Euphorbia helioscopa* L.	Dudhal	Herb	Wp, latex	Rat, mice, chicken embryo	No lesions on vital organs, and normal architecture	Oral, IV, IP,	Contact with milky sap induces skin irritation or acute inflammation in livestock. Piloerection. In severe cases, blisters may also result. Intake of plant as a whole or milky latex causes burning sensation and frothing in mouth and throat, purgation, and weakness
20	Euphorbiaceae.	*Euphorbia heterophylla* L.	Dudli booty	Herb	Wp	Cow, buffalo, sheep, goat, rat, mice,	Liver, kidney, CNS and muscles	IV, IP, oral	Livestock fed for prolonged period become weak, reduction in milk yield
21	Euphorbiaceae.	*Euphorbia hirta* L.	Lal Dudhli	Shrub	Latex	Humans, mice, rat, rabbits, dogs	Skin	IV, IP, oral	Milky juice contact with eyes and skin causes redness, severe inflammation, swelling dermatitis and boils in animals.
22	Araliaceae	*Hedera nepalensis* K. Koch	Karera	Shrub	Wp	Cow, buffalo, sheep, goat, rat, mice,	Skin, Stomach	IV, IP, oral	Dermatitis with severe inflammation, acute purgation, paralysis, death
23	Convolvulaceae	*Ipomoea carnea* Jacq.	Bilaiti aak	Shrub	Leaves	Humans, mice, rat, guinea pigs, rabbits, dogs	GIT	IV, IP, oral	Blisters in the mouth of animals, excessive salivation, acute diarrhea, shivering, inability to stand
24	Convolvulaceae	*Ipomoea purpurea* (L.) Roth	Kharpoay	Herb	Seed	Humans, mice, rat, rabbits, dogs	GIT	IV, IP, oral	Unripe seeds are purgative causing gastrointestinal irritation, diarrhea
25	Acynthaceae	*Justicia adhatoda* L.	Bahkar	Shrub		Humans, mice, rat, rabbits, dogs		IV, IP, oral	Contraction of intestine, depression, hypoglycemia
26	Verbenaceae	*Lantana camara* L.	Panjpholi	Shrub	Flowers	Cattle, goat, sheep, horse, pig, rabbit, rat, dogs, and humans	Liver, Kidney, Gall bladder, Skin,	Oral, ingestion	Hepatotoxicity, chronic cholestasis, piloerection, Photosensitization, intrahepatic cholestasis
27	Fabaceae	*Lathyrus odoratus* L.	Mattari	Herb	Wp	Sheep, goat, Rat, rabbit,	GIT	IV, IP, oral	Vomiting, nausea, debility, weakening of bones, excessive sweat, body pains leading to Lathyrism
28	Phyllanthaceae	*Leptopus cordifolius* Decne.	Kurokan	Shrub	Leaf	Humans, mice, rat, rabbits, dogs	Liver, kidney, pancreas	IV, IP, oral	Muscle weakness, piloerection, bone lesions and aneurysms, burning sensation
29	Mimosaceae	*Leucaena leucocephala* (Lam.) de Wit	Lassini	Tree	Leaves	Humans, mice, rat, guinea pigs, rabbits, dogs	Skin, GIT	IV, IP, oral	Skin allergy, loss of body hair resulting in bare patches. There is also decline in feed intake, poor weight gain and weakening of bones
30	Meliaceae	*Melia azedarach* L.	Dareek	Tree	Fruit, leaves	Rat, mice, sheep, pigs	CNS	Oral, IV, IP,	Nausea, vomiting, abdominal spasms, severe colic followed by gastroenteritis. Anxiety, restlessness, trembling of limbs
31	Fabaceae	*Melilotus indica* L.	Peeli sinji	Herb	Wp	Horse, rat, mice	Liver, blood	Oral, IV, IP,	Bleeding, liver malfunction nausea, vomiting, drowsiness
32	Apocynaceae	*Nerium oleander* L.	Kaner	Shrub	Wp, St	Wild and domestic animals, rabbit, sheep, monkey	Heart, liver, kidneys, lungs, intestine and skin	Oral, subcutaneous, steam	Piloerection, bulging of eyeballs, abdominal pain, salivation, vomiting, diarrhea, irregular heartbeat, pale color, drowsiness, tremors, seizures, coma, hepatotoxicity and nephrotoxicity, constipation, abortion, polyuria, anorexia, emaciation, leukocytosis
33	Asteraceae	*Parthenium hysterophorous* L.	Jagar booty	Herb	Wp	Domestic animals	CNS, skin	Oral	Severe allergy, itching, inflammation, rashes peeling of skin, resulting bald patches in both humans and animals Tremor, convulsions, diarrhea, dyspnea, abnormal gait anorexia.
34	Euphorbiaceae	*Ricinus communis* L.	Arind, Areni	Tree	Wp	Humans, animals, mice, rat, guinea pigs, rabbits, dogs	GIT	Ingestion, IV, IP, IM, Oral, Inhalation	Weakness, anorexia, apathy, dyspnea and moderate fever, abdominal cramps, piloerection, abortion, neurological signs, depression, acute purgation, gastrointestinal irritation
35	Asteraceae	*Senecio vulgaris* L.	Peeli jari	Herb	Wp	Domestic animals	Liver	IV, IP, oral	Jaundice, dullness, weakness, even death within a few days. In cattle, milk production also stops
36	Solanaceae	*Solanum nigrum* L.	Kayan kothi, Makoy	Herb	Leaves	Sheep, poultry, pig, cattle	Liver, CNS	Oral, subcutaneous	Dryness of throat, intense thirst, headache, nausea, vomiting, giddiness, stomach-ache, trembling of limbs, convulsions and finally death
37	Solanaceae	*Solanum surattense* Burm.f.	Neeli kandiari,	Herb	Berries	Rat, cattle, sheep, horse	Liver	IV, IP, oral	Vomiting, piloerection, swelling of face, abdominal pain, drowsiness and severe itching
38	Asteraceae	*Xanthium indicum* J.Koenig ex Roxb.	Jojra	Herb	Wp	Guinea pigs, cattle, rabbits, dogs, human, sheep, and horses	Liver, kidney	IV, IP, oral	Abdominal pain, hypoglycemia, seizures, dermatitis, nausea, vomiting, hypothermia, unconsciousness, convulsions, hepatitis, and death

Abbreviations: IP: Intraperitoneal; IV: Intravenous; IC: Intracutaneous.

### Toxic plant part (s)

The plant toxicity was observed in plants as a whole or it was restricted to some plant parts (Fig 5). The toxicity caused by whole plant was the maximum (15 spp, 39.47%), followed by leaf toxicity (12 spp, 31.58%), seed toxicity (4 spp, 7.89%), fruit toxicity (3 spp, 10.53%), latex toxicity (2 spp, 5.26%), flowers toxicity (1 spp, 2.63%) and berries toxicity (1 spp, 2.63%).

**Fig 5:** Percentage of contribution of different plant parts in livestock poisoning.

### Route of poisoning

The most toxic route of poisoning (Fig 6) was found oral (39 spp, 40.63%), followed by intraperitoneal (24 spp, 25%), intravenous (21 spp, 21.88%), ingestion (2 spp, 2.08%), subcutaneous (2 spp, 2.08%), intramuscular (2 spp, 2.08%), intracutaneous (2 spp, 2.08%), intragastric (1 spp, 1.04), inhalation (1 spp, 1.04), dermal (1 spp, 1.04), steam (1 spp, 1.04).

**Fig 6:** Different routes of administration of plant poisoning.

### Major organs affected and symptoms

The most affected organs were liver (20.41%), followed by gastrointestinal (20.341%), CNS (16.33%), skin (14.29%), kidney (12.24%), lungs (4.04%), reproductive organs (2.04%), spleen (1.75%), blood (1.75%), heart (1.75%), urinary tract (1.75%), pancreas (1.75%). The most common symptoms caused by plant poisonous were responsible were intoxication, nausea, anorexia, vomiting, salivation, emaciation, piloerection, throat blisters, diarrhea, frothing in mouth, photosensitization, irritation on nose and mouth, purgation and dermatitis followed by bloat, abdominal cramps, abortion, reduction of milk yield, adverse effect on brain, convulsions, dysphagia, poor weight gain, hallucination drowsiness, and jaundice. Other symptoms were, profuse sweating, sedation, vesication, loss of fertility, edema, lockjaw, and mouth ulceration (Table 2).

### Informant consensus factor (Fic)

The results of Fic (Table 3) show that dermatological disorders caused by plant poisoning had the highest agreement of *F*_ic_ (0.91, 17 spp), followed by the endocrine system (0.90, 2 spp), gastrointestinal (*F*_ic_ 0.82, 30 spp), neurology (0.77, 33 spp), nephrology (0.67, 2 spp), cardiovascular (0.67, 2 spp), urinary (0.67, 2 spp), respiratory (0.60, 3 spp), sexual (0.60, 5 spp) disorders. While ophthalmology (0.56, 5 spp) and death (0.50, 5 spp) had lowest number of agreements among informants. Vomiting had 40 reports, within the gastrointestinal category, dermatitis had 32 reports in dermatology, and convulsion had 20 reports in neurological signs (Table 3).

**Table 3:** Category of anomalies (Heinrich et al., 1998) [43] and their factor informant consensus (*F*_ic_) and fidelity level (Fl %) of poisonous species.

Category of anomalies	No. of reports	No. of species	*F*_ic_	Name of species	FI (%)
Dermatological	183	17	0.91	*Lantana camara*	100
				*Leucaena leucocephala*	100
				*Solanum surattense*	0.94
				*Senecio vulgaris*	0.90
				*Hedera nepalensis*	0.82
				*Ageratum conyzoides*	0.82
				*Solanum surattense*	0.81
				*Parthenium hysterophorous*	0.75
				*Dodonaea viscosa*	0.75
				*Calotropis procera*	0.71
				*Daphne oleoides*	0.71
				*Clematis grata*	0.65
				*Lathyrus odoratus*	0.55
Endocrine system	11	2	0.90	*Senecio vulgaris*	0.95
				*Ageratum conyzoides*	0.87
Gastrointestinal	164	30	0.82	*Ricinus communis*	100
				*Argemone mexicana*	0.82
				*Anagallis arvensis*	0.76
				*Achyranthes aspera*	0.71
Neurological	141	33	0.77	*Ricinus communis*	100
				*Nerium oleander*	100
				*Cannabis sativa*	100
				*Datura stramonium*	0.90
				*Datura innoxia*	0.88
				*Solanum nigrum*	0.77
				*Melia azedarach*	0.73
				*Anagallis arvensis*	0.69
				*Clematis grata*	0.65
				*Lathyrus odoratus*	0.54
				*Xanthium indicum*	0.50
Nephology	4	2	0.67	*Lantana camara*	0.90
				*Nerium oleander*	0.89
Cardiovascular	4	2	0.67	*Nerium oleander*	0.84
Urinary	4	2	0.67	*Convolvulus arvensis*	0.95
Respiratory	6	3	0.60	*Ricinus communis*	0.88
Sexual	11	5	0.60	*Cuscuta reflexa*	0.79
Ophthalmology	10	5	0.56	*Nerium oleander*	0.89
				*Datura innoxia*	0.80
				*Datura stramonium*	0.78
Death	15	8	0.50	*Anagallis arvensis*	0.83
				*Calotropis procera*	0.78
				*Ageratum conyzoides*	0.75
				*Hedera nepalensis*	0.67
				*Clematis grata*	0.59

### Fidelity level (FL)

In dermatological category (Table 3), the highly poisoned species were *Lantana camara* (*Fl*, 100), *Leucaena leucocephala* (*Fl*, 100), *Solanum surattense* (*Fl*, 0.94) and *Senecio vulgaris* (*Fl*, 0.90). For neurological disorders, *Ricinus communis* (*Fl*, 100), *Nerium oleander* (*Fl*, 100), and *Cannabis sativa* (*Fl*, 100) caused maximum poisoning. Other important species in different categories were *Ricinus communis* (*Fl*, 100), in gastrointestinal, *Lantana camara* (*Fl*, 90) in nephrology, *Nerium oleander* (*Fl*, 100) in cardiovascular, *Convolvulus arvensis* (*Fl*, 100) in urinary, *Ricinus communis* (*Fl*, 100) in respiratory, *Cuscuta reflexa* (*Fl*, 79) in sexual, and *Anagallis arvensis* (*Fl*, 83) in death.

### Hematological, biochemical and histopathological changes due to poisonous plants

We investigated the effect of poisonous plants on hematological, biochemical, histopathological and body weight changes, feed intake and indices of liver and kidney function (Table 4). The poisonous plants significantly affected various blood parameters including percentage of PCV, HB, and RBC, eosinophil, and basophil percentage, WBc count, monocytes, neutrophil, and lymphocyte counts as shown in Table 4. Predominant biochemical changes included blood serum concentrations of creatinine, total protein, globulin and cholesterol AST, ALP, uric acid, urea, GOT, and albumin (Table 4). The poisonous plants significantly affected various organs; either mildly or severely depending upon plant toxicity. Most prominent histopathological changes occur in targeted organs or systems such as CNS, GIT and skin. Common histopathological alterations include hepatization of the liver, mild pulmonary oedema, peribranchial lymphocytic infiltration of the lungs, disruption of cardiac architecture, generalized cell necrosis and erosion of the villi of the small intestine. Moreover, changes in adipose tissue, gastrocnemius muscle showed a reduction in tissue functioning, fatty degeneration, bile duct hyperplasia, and gallbladder edema (Table 4).

**Table 4:** Principal toxin, necropsy lesions and fatal dose (LD50) of the selected poisonous plants from the study area.

Sr. No	Plant Name	Toxin	Extract	Necropsy Lesions	Fatal Dose /LD_50_	Fatal period	Citations
1	*Achyranthes aspera* L.	Ecdysterone	Ethanolic	Enlargement and color changes of lungs, liver, kidney, and spleen. Emaciation of body, bronchitis, rheumatism, and dysentery	>2,000 mg/kg	60 days	[115–117]
2	*Ageratum conyzoides* L.	Pyrrolizidine alkaloids	96% Ethanolic	Hyperparathyroidism, bone tumors, rickets, hepatitis & jaundice	>10,000 mg/kg	30 days	[118, 119]
3	*Alocasia indica* (Lour.) Spach	Glycosides, glycosides	Aqueous, petroleum ether, benzene	Hepato-renal and testicular toxicity leading to infertility	144.6–400 mg/kg	15 Min	[120, 121]
4	*Anagallis arvensis* L.	Saponin, Oxalate	Alcoholic extracts	Hemorrhages of kidneys, heart, intestine, congestion of lungs, liver, and Prostate gland enlargement	1781.76 mg/kg		[37, 122]
5	*Argemone mexicana* L.	Berberine and protopine/ sanguinarine	Aqueous slurry / Root bark powder/ alkaloid	Emaciation, peritoneal edema and slightly enlarged livers with fibrinous exudate	>7000 mg / Kg.	14 Days	[96, 123]
6	*Bauhinia variegata* L	Flavonon	Methanol	Endocardial hemorrhage, gaseous distension of the gastrointestinal tract & pancreatic lesions	>2,000 mg/kg	28 days	[98, 124]
7	*Bidens bipinnata* L.	Alkaloid & steroid	Ethanol	Palpable abdominal mass, small intestinal trichobezoars at laparotomy, adenoma, and hemorrhages	>5g/kg	50 days	[115, 118, 126]
8	*Calotropis procera* Aiton	Tanines, glycosides, anthraqunions, alkaloids, flavonoids, organic acids.	Aqueous extract, Ethanolic extract	Hepatocellular necrosis, portal fibrosis, catarrhal enteritis, splenic hemosiderosis, pulmonary congestion, oedema, hemorrhages in the heart and degeneration of the renal convoluted tubules	940 mg/kg	8 weeks	[37, 127, 128]
9	*Cannabis sativa* L.	Cannabin, Cannabinol, tetrahydrocann abinol	Ethanolic, Alcoholic, Aqueous	Hemorrhages in the nervous system, emaciation, depressing effect of the poison upon vital organs	>10,000–8000 mg	5–8 Days	[28, 37, 129]
10	*Clematis grata* Wall	protoanemonin /Anemonin		Edema, reddening of the abomasum, splotchy hemorrhages on the serosa of intestines and moderate excess in abdomen fluid	1583 mg/kg	2 months	[130]
11	*Conium maculatum* L.	Coniine N-methyl coniine conhydrine		Dark petechial hemorrhages in abdominal, pectoral cavity, mesenteries blood vessels, mesenterial lymph nodes, hyperemic intestinal serosa, edematous, liver congestion, enlarged central veins of the lobules	0.1g of coniine (1 seed oral) >10000 mg/kg	30–40 min to 5 days in vary species	[129, 131–133]
12	*Convolvulus arvensis* L.	Tropane alkaloids tropine, Pseudotropine,	Ingestion, alcoholic and aqueous	Intestinal fibrosis and vascular sclerosis of the small intestine. gaseous distended intestine, congestion, oedema, and hemorrhages of many organs	165–416 mg / kg	10 days	[37, 98]
13	*Cuscuta reflexa* Decne.	Trehalose, quinolizdine	Methanolic extract	Rheumatoid arthritis, inflammation, and ulcerated nodules on oral mucosa mucocutaneous junctions of the lips, chin nose, prepuce, and anus	>2000mg/kg	21 days	[37, 134, 135]
14	*Dalbergia sissoo* Roxb	Acetylsalicylic acid	Aqueous	Myocardial infarction	>3000 mg/kg	21 days	[37, 98, 136, 137]
15	*Daphne oleoides* Schreb.	Daphnetoxin, Mezerein	Aqueous	Rheumatic pain, lumbago, bleedings	>2000mg/kg	14 days	[37, 138]
16	*Datura innoxia* Mill	Scopolamine and hyoscyamine	Methanolic crude extract	Lesions in gastrointestinal tract, hemorrhages of intestine	400 mg/kg	10 days	[37, 125]
17	*Datura stramonium* L.	alkaloids scopolamine and atropine Hyoscyamine	Ingestion, alcoholic, aqueous	Hyperthermia. Hyperirritability of CNS, lesions and hemorrhages of vitals, convulsions, coma, and death	4–5 g are fatal to a child.	7 days	[28, 37]
18	*Dodonaea viscosa* Jacq.	Pyrrolizidine alkaloids	Aqueous	Lesions in gastrointestinal track	1250 mg/kg	48 hrs.	[37, 140]
19	*Euphorbia helioscopa* L.	Non-haemolytic saponin and phasin, deoxyphorbol jatrophone-type diterpenoids euphoheliosnoi D and other toxic diterpenes	Crude ethyl alcohol	Alveolar hemorrhages, necrotic areas infiltrated by lymphocytes in lung, liver, and spleen. Proliferation of Kupffer cells, Hyaline deposits, and pinkish staining proteaceous deposits in Bowman’s capsule	1211.7 mg to 2000 mg/kg	30 to 60 days	[37, 129, 139, 141, 142]
20	*Euphorbia heterophylla* L.	Flavonoids, coumarins, saponins and tannins	Aqueous, methanolic	Enlarged liver, brain and kidneys in rats receiving high dose	2000 mg/kg.	14 days	[37, 143–145]
21	*Euphorbia hirta* L.	NR	Methanolic	Ataxia, convulsions, and paralysis	>5000 mg/kg.	14 days	[37, 96]
22	*Hedera nepalensis* K. Koch	Flavonoids, steroids, tannins, terpenoids and cardiac glycosides	Methanolic crude, aqueous extract	Shrinkage in abdominal wall, hemorrhages of vital organs, coma, and death	>5,000 mg/kg body	72 hrs.	[37, 146–149]
23	*Ipomoea carnea* Jacq.	Swainsonine, indolizidine alkaloid	Methanolic, aqueous extracts	Characteristic vacuolization of thyroid, pancreas, liver and kidneys, emaciation, thymus atrophy and spleen enlargement	>3000 mg/kg	2 hrs.	[37, 150, 151]
24	*Ipomoea purpurea* (L.) Roth	Indole alkaloids (Lysergic acid, lysergamide, elymoclavine, swansonine, and chanoclavine)	Ethanolic, aqueous	Neuronal vacuolation, endocrine dysfunction, cardiovascular, gastrointestinal, and immune disorders	>5000 mg/kg	21 days	[37]
25	*Justicia adhatoda* L.	Piperidine	Ethanolic, ether extract	Hemorrhages of vital organs	>5000 mg/kg	60 days	[58, 106]
26	*Lantana camara* L.	Lantadenes, pentacyclic triterpenoid		Jaundice, swollen liver, mottled and pale yellow to reddish yellow. icterus, moderate hydrothorax, mild dehydration	25–50 mg/kg	7 days	[25, 65, 106, 108, 152, 154]
27	*Lathyrus odoratus* L.	Lathyrogens	Ethanolic extract	Ulcer, lesion in small and large intestine,	>2000 mg/kg	22 days	[37]
28	*Leptopus cordifolius* Decne.	*Cicutoxin*	Methanolic	Lesions in gastrointestinal track	>2000 mg/kg	45 days	[27, 153]
29	Leucaena leucocephala (Lam.) de Wit	Amino acid mimosine, dihydroxypyridine (DHP)	Ethanolic extract	Hyperthyroidism, erosion of the esophageal mucosa and reticulo-rumen	>2000 mg/kg	14 days	[37, 155–158]
30	*Melia azedarach* L.	Melain	Ethanolic, aqueous	Congestion of liver and kidneys, cerebral edema & midbrain necrosis.	25–30 g/kg	3–5 days	[37, 159]
31	*Melilotus indica* L.	Coumarin, dicumarol	Ethanolic, aqueous	Hemorrhages, blood clotting	>8000 mg/kg	22 days	[173]
32	*Nerium oleander* L.	Oleandrin, Oleandrigenin, Oleandrin nerioside, oleandroside, saponins and cardiac glycosides	Aqueous, ethanolic, Methanolic,	Gastrointestinal tract hemorrhages, diarrhea, irritation, and lesions of mouth, tracheitis, congestion of lungs and death	157.37 mg / kg	4–5 days	[26, 28, 160–162]
33	*Parthenium hysterophorous* L.	Sesquiterpene lactones, parthenin	Ethanolic	Ulceration of alimentary tract, enlarged liver, emaciation, major hemorrhages, and pathological changes in kidney, liver, and skin.	676.65 mg/kg	7 days	[37, 103, 163]
34	*Ricinus communis* L.	Glycoprotein, ricin (highly toxic protein) ricinine (an irritant oil)	Ethanolic, aqueous, methanolic	Hemopericardium, hemothorax, pulmonary edema, petechial hemorrhages in the epicardium and endocardium, ecchymoses at the papillary muscles and suffusions on the intercostal muscles. Hemorrhages in the abdominal cavity, spleen and mucosa of the abomasum and small intestine	20 mg/kg	48–72 h.	[28, 104, 105, 164, 166]
35	*Senecio vulgaris* L.	Pyrrolizidine, adonifoline, senecionine	Ethanolic, aqueous	Lesions in the liver, enlarged liver and friability as well as hemorrhages.	57.3–163.3 mg/kg	46 h.	[37, 165, 167, 168]
36	*Solanum nigrum* L.	Glycoalkaloid solanine	Ethanolic & aqueous	Gastric lesions, congestion and edema of the organs, emphysema, thickening of interlobular septa, hepatocellular carcinoma	2000–5000 mg/kg	5 days	[37, 169, 170]
37	*Solanum surattense* Burm.f.	Solanine A, alkaloids, flavonoids, tannins, sterols and saponins	Alcoholic	Liver malfunctioning, thickening of blood vessels and gastrointestinal disorder	2000 mg/kg	5 days	[37, 171]
38	*Xanthium indicum* J.Koenig ex Roxb.	glycoside carboxyatractyloside	chloroform	Ascites with fibrin strands, enlarged, congested and friable livers with accentuation of lobulation on the capsule	3000 mg/kg	6–92 hrs.	[172]

### Fatal period and necropsy lesions

Literature study revealed that LD_50_ of poisonous plants were investigated concerning the toxicity of the active principle of the poisonous plant in the laboratory animals and grazing animals were depending upon the exposure of toxins and their route of administration (Table 5). Our results concerning the LD_50_ of the active principle of poisonous plants revealed that the doses of the LD_50_ were different for animals under varying environmental conditions. There is dearth of literature regarding LD_50_, fatal periods and necropsy lesions of poisonous plants growing under local environmental conditions in AJK (Table 5).

**Table 5:** Plant-based hematological, biochemical and histopathological observations in animals.

Sr. No	Plant Name	Hematology	Biochemical changes	Histopathology
1	*Achyranthes aspera* L.	Slightly increase of RBCs, increase in number of monocytes and eosinophils, decrease in number of Neutrophils and lymphocytes	Urine thickness, increased levels of SGPT, SGOT, SALP, GGT, bilirubin, and LPO.	High fibrocytes, mild kidney and spleen damage
2	*Ageratum conyzoides* L.	No significant changes in haematological parameters including red blood cells, WBC, and platelets.	Low serum, ALT, AST, LDL, high density lipoprotein, fatty acids and urea	Cell damage, over production of tissues
3	*Alocasia indica* (Lour.) Spach	RBCs, Hb, total protein, albumin and globulin significantly decreased,	AST, ALT, GGT, LDH, urea, creatinine, total lipid, and cholesterol significantly increased. Low serum level in low testosterone, sperm abnormalities, γ-GT, and total bilirubin reduced.	Changes in liver architecture, liver cellular degeneration, necrosis, hepatotoxicity, and apoptosis of liver. Kidney tubular necrosis, glomerular shrinkage and atrophied glomerular tuft of capillaries.
4	*Anagallis arvensis* L.	Severe anemia, decreased hemoglobin concentration, packed cell volume and erythrocyte count and no changes in WBC count	Significantly increased urea and creatinine levels.	Chronic interstitial pneumonitis, alveolar emphysema, bronchitis, hyperplasia, hepatocytes swollen, prostatitis, heart -mild peri-vascular edema, kidney congestion, occasional hemorrhage, necrotic changes
5	*Argemone mexicana* L.	Elevated Eosinophils count, Neutrophils, HGB, RBCs & WBCs Reduction in lymphocytes	Significantly increase in total protein and albumin	Alterations were limited to catarrhal enteritis in turkey
6	*Bauhinia variegata* L	Reduction in lymphocytes, monocytes and hemoglobin concentration, No changes in other hematological parameters	Decrease in AST, blood glucose levels. Lipid profile, cholesterol, triglyceride, Total proteins, and albumin no significant changes in normal levels.	Minimal changes in liver, kidney parenchyma, focal congestion of blood vessels and cellular swelling with granular cytoplasm. stomach, spleen, pancreas, adrenal, lungs, heart, brain, ovaries, and testicles did not show any structural changes
7	*Bidens bipinnata* L.	Significantly increase hemoglobin	Significantly elevated glucose level, decrease in proteins and the albumin	No significant microscopic lesions observed in the liver, spleen, lung, kidney, and brain
8	*Calotropis procera* Aiton	Significantly increased eosinophil, basophil, hemoglobin, PCV and platelet values in blood leading to normocytic normochromic anemia	High ALT, AST, and ALP in serum, increase concentration of ammonia, sodium, potassium, creatinine. Decreased blood protein level and calcium	Mild pulmonary oedema, lungs infiltration, hepatization of liver, disruption of cardiac architecture, cell necrosis and erosion of villi in small intestine.
9	*Cannabis sativa* L.	Granulocytes, lymphocytes, WBC, RBC, monocytes, Hemoglobin, packed cell volume and platelet levels significantly reduced (p<0.05)	AST and ALT, Albumin, Globulin, Total protein, Conjugated bilirubin while Total bilirubin, unconjugated bilirubin concentration significantly increase in serum	Inflammation, degeneration and necrosis in adipose tissue, gastrocnemius muscle showed a damage in tissues
10	*Clematis grata* Wall	Significantly did not alter RBC, Hb, PCV, MCV, MCH, MCHC and RCDW levels but increase neutrophils, monocytes, eosinophils and basophils levels, Reduction in WBC, platelet, lymphocytes, uric acid, triacylglycerol	significantly did not alter the liver-and kidney-body weight ratio, conjugated bilirubin, total protein, globulin, sodium, potassium, chloride, inorganic phosphorus, calcium ions, LDL-C, levels but increase albumin, urea, HDL-C, LUC, AST, GGT, ALT, ALP	severe infiltration of inflammatory cells, with disruption and loss of articular cartilage
11	*Conium maculatum* L.	Significant increases in blood glucose	Significant increases in blood BUN and SGOT and SGPT, loss of microsomal cytochrome P-450 and benzphetamine N-demethylase activity	Hepatocytolysis, nuclear degeneration, pyknosis, cloudy swelling, sinusoids liver, proliferated endothelium of glomeruli, hemorrhage in glomeruli and interstitial, swelling of kidney, atrophy stomach mucosa, congestion duodenum
12	*Convolvulus arvensis* L.	Decrease Hb, PCV and RBC count and anemia	Elevation of enzymes indicating liver and kidney dysfunction	Gaseous distended intestine, congestion, oedema, and hemorrhage of many organs
13	*Cuscuta reflexa* Decne.	Significantly improved the levels of neutrophil, lymphocyte, hemoglobin, RBC, and platelet,	NR	active follicular proliferation, increased tissue permeability
14	*Dalbergia sissoo* Roxb	Haematological parameters were not affected	Alanine aminotransferase, aspartate aminotransferase and creatinine were not affected	Changes in the epididymis and testis, degeneration of seminiferous tubules
15	*Daphne oleoides* Schreb.	Decrease RBC count, Hb, PCV and anemia	Significant increase in cholesterol, triglycerides, ALT, AST, ALP	Lymphocytic leukemia, infiltration of lymphocytes, monocytes, neutrophils
16	*Datura innoxia* Mill	Significantly decrease in platelets, RBCs, hemoglobin, hematocrit	Change in lipid composition, enzymes of reproductive organs, increase in AST, ALT, LDH, GGT	Change in liver and renal tissues
17	*Datura stramonium* L.	Significant decrease in RBCs, hemoglobin, hematocrit, and platelets levels	Significant increase in AST, ALT, LDH, GGT, PLA, urea and creatinine Na+ and K+ concentrations	High degree of vacuolization and inflammation in liver and the same up to lesser extent in kidney
18	*Dodonaea viscosa* Jacq.	Significantly improve the level of these cells’ RBCs, WBCs, and Platelets	Significantly restore the level of hepatic enzymes ALP, AST ALT, Direct bilirubin, total protein, and liver antioxidant enzymes SOD, GPx, and CAT	Fibrosis and vascular irregularities, for instance, liver sinusoids alteration and central vein congestion
19	*Euphorbia helioscopa* L.	Significantly elevate in RBCs, hemoglobin, hematocrit and platelets levels	Decrease in cholesterol, triglycerides, LDL and VLDL levels of latex and leaves with methanol extract-treated animals, with respect to control indicating plant’s hypolipidemic effect	Mildly congested central veins, mild inflammation, and sinusoidal, intense diffused infiltration of the sinusoid by dense inflammatory cell aggregates
20	*Euphorbia heterophylla* L.	Significant increase in hematocrit, hemoglobin, RBC, platelets and mostly decreased white blood cells	Significant elevation in AST, ALT, ALP and Decrease in cholesterol, triglycerides, LDL and VLDL	Mild inflammation, portal congestion and sinusoidal, intense diffused infiltration of the sinusoid by dense inflammatory cell aggregates and mildly congested central veins
21	*Euphorbia hirta* L.	Changes in haemoglobin, hematocrit, platelets and blood cell count	Significantly change in kidney and liver ALT, AST, total protein, globulin, and albumin	Normal structure and absence of any gross pathological lesion in rats
22	*Hedera nepalensis* K. Koch	Significant increase in hematocrit, hemoglobin, RBC, platelets and mostly decreased white blood cells	Significant decrease in GGT, ALP, creatinine, total protein, total bilirubin, cholesterol, triglyceride, glucose level. ALT, and albumin level increased at the dose rate of 400 mg/kg body weight in rabbits	Liver and kidney showed mild to severe pathological lesion in a dose dependent manner.
23	*Ipomoea carnea* Jacq.	Decrease in packed cell volume, hemoglobin, and total erythrocyte count	Significantly change in kidney and liver ALT, AST, total protein, globulin and albumin	Changes in hepatic cells, inflammatory cells
24	*Ipomoea purpurea* (L.) Roth	Significantly alteration in hematology	Significantly increase in globulin, AST, ALP, protein, albumin, and bilirubin	Morphological changes in hepatic and pancreatic cells
25	*Justicia adhatoda* L.	Higher dose 5g/kg then increased RBC, hemoglobin, and platelet	Increased activity of liver superoxide dismutase (SOD)	Liver and kidney showed mild to severe pathological lesion in a dose dependent manner
26	*Lantana camara* L.	Increased blood clotting time, leukocyte count and hematocrit values, progressive decrease in packed cell volume, hemoglobin, and total erythrocyte count	Increase in total bilirubin, phylloerythrin levels, AST, ALP, GLDH, serum total protein, albumin, and globulin, decrease in albumin/globulin ratio	Fatty degeneration, bile duct hyperplasia, gall bladder edema, degeneration of parenchymal cells and portal fibrosis, hemorrhages of inter-sinusoidal spaces, coagulative necrosis, cirrhosis, and proliferation of bile ductulus of kidney and liver
27	*Lathyrus odoratus* L.	Decrease in packed cell volume, hemoglobin, and total erythrocyte count	Significantly increase in globulin, AST, ALP, protein, albumin, and bilirubin	Infiltration of inflammatory cells, fibrosis, necrosis, cell injury
28	*Leptopus cordifolius* Decne.	Significantly reduced blood glucose level in mice.	Significant elevation in total cholesterol, triglyceride, LDL, HDL, SGPT, SGOT, ALP and creatinine. significantly reduced antioxidant enzymes, like CAT, POD, SOD levels, and elevated the action of reactive oxygen species	Morphological changes in hepatic and pancreatic cells
29	Leucaena leucocephala (Lam.) de Wit	Significant decrease in hematology RBC, hemoglobin and platelet	Increase in bilirubin, AST, ALP, protein, albumin, and globulin	Atrophic and germ cell degenerating seminiferous
30	*Melia azedarach* L.	Significant decrease in RBC count, hemoglobin and platelet	Significantly increase in AST, ALT, ALP, LDL.HDL, albumin, and bilirubin	Infiltration of inflammatory cells, fibrosis, necrosis, cell injury
31	*Melilotus indica* L.	Decrease in packed cell volume, hemoglobin, and total erythrocyte count	Significantly increase in globulin, AST, ALP, protein, albumin, and bilirubin	Changes in hepatic cells, nephritis, and pancreatic cells
32	*Nerium oleander* L.	Significant variations in RBCs, Hb, Hct, MCV, lymphocyte, neutrophil, monocyte and eosinophil count	Significantly increase ALP, LDH, total protein, urea, creatine kinase (CK), and creatinine	Myocardial degeneration, hemorrhages, multifocal coagulative necrosis of the cardiac muscle fibers, and severe and diffuse enteritis, diffuse passive hyperemia and mild, multifocal hemorrhages, hepatic necrosis, widening of sinusoidal spaces and mild vascular damage
33	*Parthenium hysterophorous* L.	Significantly decreased MCH, RBC, Hemoglobin, and platelet, haematocrit, WBC count significantly increased in Labeo Rohita.		Inhibition of key cellular enzymes like succinate dehydrogenase, phosphofructokinase, glucose -6- phosphatase, glutamate oxaloacetate transaminase, acid and alkaline phosphatases	Severe degenerative changes in the liver and kidney due to the presence of a cyclopentene group, which can cause chromosomal damage in animal cells, uncouple phosphorylation and inhibit key cellular enzymes, allergenic rhinitis, erythema, edema
34	*Ricinus communis* L.	Significant reduction in the PCV, Hb, total RBC, MCH, significantly increased WBC count, neutrophil/lymphocyte, monocyte/lymphocyte, cholesterol, and triglyceride	Significantly did not change in Albumin Cortisol, Total serum bilirubin and ALT, but AST value was increased, while Adenosine phosphatase (AP) value was deceased.	Multifocal coagulative myocardial necrosis with the presence of mononuclear cell infiltration and varying degrees of bleeding between cardiac muscle fibers, mild edema in small intestine, inflammatory cell infiltration.
35	*Senecio vulgaris* L.	Significantly decrease in RBCs, Hb, Hct, MCV, lymphocyte, neutrophil, monocyte and eosinophil count	Increase in the serum activity of ALT, ALP, GOT, AST and bilirubin	Degeneration, necrosis, fibrosis in cells of liver, heart, kidney, and brain
36	*Solanum nigrum* L.	Significantly decreased RBC, platelets count, PCV and Hb levels. However, it increased WBC count.	No significant changes in AST, ALT, ALP, Nitric oxide, lipid peroxidation, glutathione peroxidase, alkaline phosphatase, and total bilirubin but increased activity of glutathione peroxidase.	Showed no pathological effect on the morphology of the liver, spleen, heart and kidney of the rats.
37	*Solanum surattense* Burm.f.	Mild leukocytosis	Increase in liver enzymes	Hepatic congestion, necrosis, degeneration, and cell injury same in kidney and brain
38	*Xanthium indicum* J.Koenig ex Roxb.	Significantly reduction in RBC, hemoglobin, hematocrit (HCT), MCV, platelets, WBC (total), and WBC (differential).	Significantly increase in liver enzymes AST, ALT, ALP, GGT, hypoglycemia, total bilirubin, direct bilirubin, hypoalbuminemia, cholesterol, creatinine, and triglycerides with leukocytosis by neutrophilia with regenerative left shift.	Acute hepatic congestion and hemorrhage, centrilobular hepatocyte necrosis, discoid lysis of skeletal and cardiac muscle fibers, no histopathological abnormalities

### LD_50_

*Ricinus communis* with reported LD50 (<20 mg/kg) was the top-ranked poisonous plant followed by *Lantana* camara and *Justicia adhatoda* (25–50 mg/kg), *Nerium Oleander* (157.37 mg/kg), and *Datura innoxia* (400 mg/kg). Rest of the plants showed >1000 LD_50_. Based on the informant score, *Ricinus communis* was found with highest level of toxicity (84/100), trailed by *Lantana* camara (82/100), *Nerium Oleander* (78/100), *Datura innoxia* (74/100), and *Leptopus cordifolius* (70/100) as depicted in Table 6.

**Table 6:** The top ranked poisonous plants based on their LD50 and respondent scores.

Plants	LD_50_	Respondent (R1-10)										Score	Percentage	Rank
		R1	R2	R3	R4	R5	R6	R7	R8	R9	R10			
*Ricinus communis*	<20 mg/kg	8	10	8	9	7	9	7	8	10	8	84		1^st^
*Lantana camara*	25–50 mg/kg	9	9	10	8	8	7	8	9	7	7	82		2^nd^
*Nerium oleander*	157.37 mg / kg	10	8	8	7	6	7	8	8	7	9	78		3^rd^
*Datura stramonium*	400 mg/kg	7	8	8	7	9	9	8	7	5	6	74		4^th^
*Leptopus cordifolius*	>2000 mg/kg	7	9	5	5	7	6	8	6	9	8	70		5^th^
*Solanum surattense*	>2000 mg/kg	8	8	7	8	5	4	3	7	5	8	63		6^th^
Euphorbia helioscopa	1211–2000 mg/kg	5	5	6	6	5	8	6	6	6	5	58		7^th^
*Dodonaea viscosa*	1250 mg/kg	5	6	7	7	5	5	8	3	4	5	55		8^th^
*Justicia adhatoda*	25–50 mg/kg	7	4	5	5	6	4	5	6	5	6	53		9^th^
*Bauhinia variegata*	>2000 mg/kg	6	5	4	5	3	5	4	4	4	5	45		10^th^

## Discussion

The present study is the first detailed report on toxic effects of poisonous plant on livestock and experimental animals. The data was gathered from extensive surveys and literature reviews on poisonous plants of AJK. A total of 271 informants belonging to various professions and age groups were interviewed to attain the information regarding toxicity, effected organs, necropsy lesions, fatal dose, fatal period, predominant toxic chemicals induced in body, clinical symptoms, biochemical changes, hematology, and histopathology. The authenticity of the data collected from local people was tested by using standard indices. It has been reported that plant poisoning occurs more often accidentally or under water deficit conditions (drought), fire, overstocking and trample of the grazing land [52]. Accidental poisoning in humans might occur because of contaminated food by plant poisoning and confusing poisonous with edible plants [15, 53, 54], medicinal use of toxic plants [55], fatal cases most commonly occur without diagnosis [56] or documentation [57]. Even the smaller quantity of poisonous plants poses deleterious effects in the body of any animal [58] and could be lethal because they contain powerful toxic ingredients including phytochemicals [29, 30]. These toxic ingredients produce harmful effects by harming the cell protoplasm and these effects might be immediate or accumulative [59] and their concentration differs from plant to plant and seasonal changes. The important poisonous plants produced different ailments and their toxic components as already been described in earlier studies [15, 32, 60–66].

Family is an important mean for classification of different plant species in order to determine the efficacy of plant species to local people [67]. Same is also true for the toxicity of poisonous plants [68]. Asteraceae, Solanaceae, Fabaceae, and Euphorbiaceae were reported among the most important families containing toxic plants. The plants of these family are mainly responsible for plant poisoning and have been documented earlier by many researchers [32, 68–71]. These families are toxic because of the presence of toxins like alkaloids [72–74], glycosides [38, 75–77], saponin [78, 79] teroids [80–82], and other cyanogenic glucosides and glucosinolates [83–85].

We found that whole plants and leaves were the most toxic plant parts. Leave are physiologically most active plant parts, and they are consistently reported to be used for grazing and medicinal purposes [41]. The reason behind this is that leaves are nutritional very rich plant part and are easily chewed or ingested by the animals compared to seeds and fruits [19].

We reported in our study that most of the toxicity in livestock was caused by the plants which were rich is alkaloids, glycosides, saponin, and cyanogenic compounds. Alkaloids are extremely poisonous to animals which can affect nervous system and cause liver damage [86]. Most prominent symptoms induced by alkaloids depression, abortion, and trembling, vomiting paralysis leading to death [73, 87, 88]. Whereas, glycosides may cause paralysis, excitement, staggering, prostration, gasping, convulsions, blindness leading to coma and death; nitrogenous compounds cause depression, abortion, hemorrhages which can even leads to coma and death [89–92]. Saponins may cause inflammation of skin, liver damage, restlessness, itching and necrosis of skin which might leads to death due to kidney failure [93]. Herbs and shrubs were the most dangerous species found, as these are frequently available to cattle, whereas tree fodder is provided to them in times of scarcity when herdsmen ascend and remove branches off trees [60, 94, 95].

The current study revealed various important categories of disorders caused by poisonous plants with high Fic scores. These mainly include dermatological, endocrine, gastrointestinal, neurological disorders. Factor informant consensus (Fic) provides a powerful analytical tool to select illness categories [49]. Therefore, the dermatological disorders with maximum Fic value (0.91) were key ailments caused by plant poisoning trailed by endocrine and gastrointestinal disorders. Fic further validated the deleterious effects to animals affected by consumption of the poisonous plant.

Dermatological and gastrointestinal problems are the animal’s initial response to the poisons of poisonous plants, and if they are not diagnosed and treated in a timely manner, they might lead to death [37]. Plant poison may cause piloerection and diarrhea as first appearance of dermatological and gastrointestinal sign when used, but toxin nature and effects differ significantly. Plant with high FL values such as *Lantana camara*, *Leucaena leucocephala*, *Nerium oleander*, *Ricinus communis*, and *Cannabis sativa* have been reported to cause dermatitis and affect gastrointestinal tract in some other studies [96–99]. *Lantana camara* spread poisoning sporadically in most of the livestock and cause high mortality and loss of productivity when ingested accidently [65]. Most of the animals are sensitive to *Nerium oleander* and principal toxin oleandrin directly cause cardiotoxicity and CNS disorders [100], and cardiac glycosides sometimes have fatal side effects, including gastric problems, enhanced respiration, and nervous disorder [56].

Despite the presence of mimosine in the leaves, *Leucaena leucocephala*, a high-quality ruminant feed, is necessary for livestock production in the tropics. However, high levels of mimosine might have a negative impact on animal wellbeing. Change in weight gain and weight loss, increased salivary flow, esophagus ulcers, increased thyroid, loss of hair, delayed growth, and oral ulcers all are symptoms of *L*. *leucocephala* poisoning [101]. The toxicological profile of *Cannabis sativa* intoxication is directly related to the proportion between the concentrations of ingested sample and mainly symptoms are related to the central nervous system [102].

*Ricinus communis* was reported highly poisonous plant based on LD50. The high toxicity in *R*. *communis* may be due to presence of proteaceous glycoprotein and ricin which affect the hemoglobin level in animals and have deleterious impact on cardiac fibers and intestinal mucosae [28, 103–105]. Other plants with high LD50 were *Lantana camara*, *Justicia adhatoda* and *Nerium oleander*. The lantadenes and pentacyclic triterpenoid compounds are responsible for poisoning in [65, 106]. These toxins directly increase the level of bilirubin in blood and cause severe damage to liver in animals [65, 106–108]. The level of toxicity in plants vary depending on the ecological conditions of the area. Other important factors are potency and concentration of the toxicants in plant part eaten by the animals, route of exposure, dose, and overall sensitivity of animals to toxicant. According to the reported literature, *Dodonaea viscosa* and *Justicia adhatoda* are highly toxic to the livestock but based on the respondent’s experience and observations, these plants were reported as less toxic. This difference in the claims can be linked to the fact that concentration of toxics may vary in different parts of the plants depending on the geographic location, growing condition, and time of year. For example, all parts of the *N*. *oleander* are toxic but in majority of the plants, seeds and unripen fruits are much toxic compared to the leaves and ripened fruits [109].

The current study reported that poisoning in plants undertaken brought significant hematological, biochemical, histopathological changes in livestock. The poisonous plants significantly affected various blood parameters including percentage of PCV, HB, RBCs, and predominant biochemical changes involved change in blood serum values. Most prominent histopathological changes include microscopic lesions in targeted organs such as CNS, GIT, skin, hepatization of the liver, mild pulmonary, and oedema. Administration of *L*. *camara* lantadenes caused acute liver and renal toxicity, leading in body weight loss and toxicity, with the highest dose (24 mg/kg bw) causing the most lesions and the lowest dose (6 mg/kg bw) causing the least [110]. Oleandrin present in *N*. *oleander* revealed significant increases in the red and white blood cell counts, haemoglobin concentration and caused interstitial pneumonia in the lungs and degeneration and necrosis of muscles fibers in the heart [23]. The ricin is the toxic principle in *Ricinus communis* in leaves and seeds [111]. Hemopericardium, hemothorax, respiratory failure, pericardial effusion internal bleeding in the epicardium and endocardium, ecchymoses at the papilla, and suffusions on the intercostal muscles are among the visual abnormalities observed. Hemorrhages in different organs, myocardial necrosis, inflammatory cell infiltration [103], with increased AST and decreased AP in the blood is often reported [112]. The higher level of alkaloids such as atropine, hyoscamine and scopolamine present in *Datura stramonium* triggered tachycardia, difficulty in breathing, convulsions and a decrease in locomotor activity, significant decline in RBCs and HB in blood, increased level of AST and ALT, diarrhea, and inflammation of liver [113, 114].

### Conclusion

The present study is the first comprehensive report with emphasis on the poisonous plants which are great threat to the livestock in Azad Jammu and Kashmir. Even the smaller quantity of poisonous plants poses harmful effects on the health status of livestock. A total of 38 species found in AJK were reported, which are economically important to nomads and domestic population as they cause huge economic losses domestically. Our findings show that poisonous plant awareness is less prevalent in AJK’s remote regions than knowledge of other medicinal plants. Toxic compounds such as glucosides and alkaloids produced by these plants are key factors for plant poisoning in livestock. The digestive, neurologic, and skin problems persist more often in livestock due to plant poisoning. More research is needed to validate traditional information about toxic plants in appropriate experimental settings, as well as to discover the identity of toxic phytochemicals linked with poisonous plants. Furthermore, future studies should evaluate the therapeutic aspects of these dangerous plants so that molecules of pharmacological interest with potential application in the treatment of cattle and human diseases can be discovered.

## Abbreviations

OECD: Organization for Economic Cooperationand Development
HEXSR: Hexane soluble fraction of Xanthium strumarium root
CEXSR: Chloroform soluble fraction of Xanthium strumarium root
ALP: Alkaline phosphatase
AST: Aspartate aminotransferase
ALT: Alanine aminotransferase
DC: Differential leukocyte count
